# Obesity Accelerates Leukocyte Telomere Length Shortening in Apparently Healthy Adults: A Meta-Analysis

**DOI:** 10.3389/fnut.2022.812846

**Published:** 2022-05-26

**Authors:** Sheida Khosravaniardakani, Dmitry Olegovich Bokov, Trias Mahmudiono, Seyedeh Sedigheh Hashemi, Negin Nikrad, Shadi Rabieemotmaen, Mahdieh Abbasalizad-Farhangi

**Affiliations:** ^1^Student Research Committee, Shiraz University of Medical Sciences, Shiraz, Iran; ^2^Institute of Pharmacy, Sechenov First Moscow State Medical University, Moscow, Russia; ^3^Laboratory of Food Chemistry, Federal Research Center of Nutrition, Biotechnology and Food Safety, Moscow, Russia; ^4^Department of Nutrition, Faculty of Public Health, Universitas Airlangga, Surabaya, Indonesia; ^5^Department of Nutrition, School of Health and Nutrition, Bushehr University of Medical Sciences, Bushehr, Iran; ^6^Student Research Committee, Tabriz University of Medical Sciences, Tabriz, Iran; ^7^Department of Biology, East Tehran Branch, Islamic Azad University, Tehran, Iran; ^8^Department of Community Nutrition, Faculty of Nutrition, Tabriz University of Medical Sciences, Tabriz, Iran

**Keywords:** telomere length, obesity, systematic literature search, meta-analysis of hypothesis, adult

## Abstract

**Background:**

Shorter telomere length is associated with numerous comorbidities. Several studies have investigated the role of obesity in telomere shortening. In the current systematic review and meta-analysis, we summarized the results of studies that evaluated the association between obesity and telomere length.

**Methods:**

A systematic search from Scopus, PubMed, Embase, and ProQuest electronic databases up to 19 March 2021 without language restriction was performed and after data extraction and screening, 19 manuscripts were eligible to be included in the final meta-synthesis.

**Results:**

The highest category of telomere length was associated with an approximate 0.75 kg/m^2^ reduction in body mass index (BMI; WMD = −0.75 kg/m^2^; CI = −1.19, −0.31; *p* < 0.001; *I*^2^ = 99.4%). Moreover, overweight/obese individuals had 0.036 kbp shorter telomere length compared with non-overweight/obese adults (WMD = −0.036; CI = −0.05, −0.02; *p* = 0.030; *I*^2^ = 100%). According to the results of subgroupings, continent, age, and sample size could be possible sources of heterogeneity.

**Conclusion:**

From the results, it was clear that obesity was associated with shorter telomere length. Because of the observational design of included studies, the causality inference of results should be done with caution; thus, further longitudinal studies are warranted for better inference of causal association.

## Introduction

The concept of “telomeres” was first introduced by McClintock et al., who determined that the ends of the chromosome are responsible for the stability and integrity of the chromosome, and they named it “telomere” (1). Thus, the telomere, at the end of the chromosome, is composed of thousands of tandem repeats of the TTAGGG nucleotide sequence (2, 3). Telomeres are crucial factors in the genome’s structural integrity and protection of chromosomes from erosion (4, 5). This erosion takes place in every cycle of replication, and the consequent telomere shortening is a leading cause of cellular apoptosis (6, 7), a process that is triggered by inflammation and oxidative stress (8, 9). Telomere shortening is associated with cardiovascular events, stroke, type 2 diabetes, and a higher mortality rate (10). Several lifestyle-related factors are associated with telomere shortening like smoking (11–13), alcohol intake even in minor amounts (14, 15), low physical activity (16, 17), and high-fat diets (18, 19) that trigger telomere shortening. Obesity is a well-known risk factor for many age-related comorbidities and directly increases the risk of oxidative stress and inflammation (20, 21). Several previous studies have introduced obesity as a leading cause of telomere shortening (22–24). For example, in a population-based study by Chen et al. (2014) (5), obesity was associated with shorter telomere length among 3,256 American-Indians aged 14–93 years (5). This association possibly is mediated by adiposity, and higher body fat mass is mainly responsible for reducing telomere length; abundant evidence suggests that reduced adiposity through caloric-restriction interventions will be helpful in maintaining telomere length or increasing it (25, 26). In a study of 42 obese individuals after 6 months of bioenteric intragastric balloon (BIB) placement for weight loss, a remarkable increase in telomere length after the intervention was reported (from 3.58 ± 0.83 to 5.61 ± 3.29 kbp, *p* < 0.001) (27). Although the association between obesity and telomere length is reported in several studies, making a conclusion about this association is not possible unless performing a summarized analysis to confirm this association; therefore, in the current meta-analysis, we summarized the results of cross-sectional studies that evaluated the association between obesity measures (e.g., body mass index, BMI) and telomere length in adults.

## Materials and Methods

The results of the current study were reported according to Preferred Reporting Items for Systematic Reviews and Meta-Analyses (PRISMA) (Supplementary Table 1) (28). In addition, the 12-item PRISMA extension checklist was used for abstract writing (29). The study protocol was registered in the International Prospective Register of Systematic Reviews system (PROSPERO) with the identification number CRD42021243523.

### Search Strategy

Through a systematic search from Scopus, PubMed, Embase, and Proquest electronic databases, a total of 6,807 articles that evaluated the association between obesity and telomere length up to 19 March 2021 were retrieved. No language restriction was applied. A hand-searching from reference lists of all relevant articles, systematic reviews, and meta-analyses was also done to find any possible missed publication. The search strategy was created with a combination of the Medical Subject Headings (MeSH) terms from the PubMed database and free-text words. The search strategy for PubMed is shown in Supplementary Table 2.

### Selection of the Studies

Our search results from the Scopus, PubMed, Embase, and ProQuest electronic databases provided a total of 6,807 articles. The retrieved articles were imported into EndNote software, and duplicate articles were removed. After duplicate removal (e.g., 2,446), a total of 2,156 articles have remained. The remained articles were checked by 2 investigators (MAF and TM). In total, 2,137 articles were excluded because of irrelevant design, subject, languages other than English, other age groups, being conferences, congresses, and seminars, being in other chronic diseases like several types of cancers, HIV, Cushing’s syndrome, schizophrenia, chronic kidney disease, cystic fibrosis, etc. Some of the excluded studies did not evaluate the requested association of studied parameters. Any discrepancies between reviewers were resolved by discussion with a third investigator (DOB). Consequently, 19 manuscripts were included in the final meta-synthesis (Figure 1).

**FIGURE 1:** Study flowchart.

### Inclusion and Exclusion Criteria

In the current systematic review and meta-analysis, inclusion criteria were as follows: (1) cross-sectional studies, (2) the studies that evaluated the relationship between telomere length and overweight/obesity measurements as BMI or fat mass, (3) the studies that were conducted among adults (>18 years), and (4) studies that provided the odds ratio (OR) of the association between telomere length and overweight/obesity measurements or those which provided mean ± standard deviation (SD) of BMI or fat mass. Interventional studies, reviews, case reports, and case series, experimental and *in vitro* studies, short communications, letters to editors, and studies that examined the relations other than the relationship between telomere length and obesity measures or those which did not provide OR or mean (SD) of BMI were excluded.

### Data Extraction and Quality Assessment of Included Studies

Data extraction was performed independently by two authors (MAF and TM), using a standard Excel extraction datasheet. First author and journal name, country, year of publication, the age range of participants, study design, the total number of participants, adjusted covariates, gender, setting, telomere length measurement tools, and main results of the studies were extracted from all of the selected articles. The methodological quality of included studies was assessed using the Agency for Healthcare Research and Quality (AHRQ) checklist (30). The items were scored as follows: score of “1” and “0” for “YES” and “NO” or “UNCLEAR” answers, respectively. The final quality scores were low quality = 0–3; moderate quality = 4–7, and high quality ≥ 8. There were no quality criteria for the inclusion of the studies in the current meta-analysis (Supplementary Table 3).

### Statistical Analysis

Data analysis was performed by STATA version 13 (STATA Corp, College Station, TX, United States). The *p*-values less than 0.05 were considered statistically significant. Generally, in the two-class meta-analysis, two approaches were identified: first, the studies that evaluated the association between odds of overweight/obesity and telomere length; and second, the studies that reported the comparison of relative telomere length [mean (SD)] in those with the highest vs. the lowest BMI. Therefore, the OR and confidence interval (CI) or the mean and SD of the variable was used to calculate the unstandardized effect size calculated by a pooled estimate of OR or weighted mean difference (WMD) with a 95% CI. When the data of the exposure of variable in the groups instead of OR were provided, we calculated the prevalence ORs (PORs) as suggested by Pearce N as the best approach for measuring effect size in a prevalence study (31) as follows: $POR=\left[\frac{P1}{1-P1}\right]/\left[\frac{P0}{1-P0}\right],$ where P0 and P1 are the prevalence in exposed and non-exposed groups, respectively. When the median and range were reported instead of mean and SD, the method of Hozo et al. (2005) (31) was used considering the median values as the best estimate of mean when the sample size of the study was more than 25 and the SD was calculated as follows: $S^{2}\approx (\frac{1}{12}(\frac{{\left(a-2m+b\right)}^{2}}{4}+{\left(b-a\right)}^{2}$). For missing SDs, the method of Walter and Yao was used as SD = (*b* − *a*)/4. This method was the improved version of the “range” method (33, 34). If the number of participants in categories was not available, it was assumed that an equal number of participants in each category was allocated. For measurement of the heterogeneity between studies, Cochran’s *Q* and *I*^2^ tests were used considering no heterogeneity for *I*^2^ < 25%, moderate heterogeneity for *I*^2^ = 25–50%, and large heterogeneity for *I*^2^ > 50% (35). For significant heterogeneities of either the Q statistic with *p* < 0.1 or *I*^2^ > 50%, the random-effects model was used (36). Subgrouping was also performed to identify the source of heterogeneity. Begg’s funnel plots followed by Begg’s adjusted rank correlation and Egger’s regression asymmetry tests were used for the assessment of publication bias.

## Results

### Characteristics of the Included Studies

Totally, 12 studies were included in the first, two-class meta-analysis of the comparison of BMI between the lowest and the highest leukocyte telomere length (LTL) categories (4, 5, 37–46). This meta-analysis included a total number of 35,655 adults in the age range of 18–80 years old. Of 12 included studies, six studies reported significantly lower BMI in the highest vs. the lowest LTL categories (4, 5, 38, 42, 43, 46); in three studies (37, 39, 40), BMI in the highest LTL was non-significantly lower than the highest category. In the study by Zalli et al. (2014) (45), no significant difference in BMI between LTL categories was reported; in two studies, BMI in the highest LTL categories was either significantly or non-significantly higher than the lowest category (41, 44). Only the study by Hardikar et al. (2015) (44) was performed in patients with Barrett’s esophagus, whereas other studies included apparently healthy adults. All of the studies had a cross-sectional design, and LTL was assessed with quantitative polymerase chain reaction (qPCR). Except for the study of Julin et al. (2017) and Cassidy et al. (2010) (4, 43), that was performed in men and women, respectively, the other studies were performed in combination of both genders. Eight studies were performed in the United States (4, 5, 40–44, 46), one in the United Kingdom (45), one in China (37), one in Lebanon (38), and one in Australia (39). Only, two studies reported the comparison of fat mass between different LTL categories (38, 42), and therefore, the meta-analysis was not performed. The comparison of LTL between obese/overweight, or non-obese/non-overweight was reported in seven studies and presented in the second two-class meta-analysis. The meta-analysis is composed of 32,467 participants, and all of the participants were apparently healthy individuals aged between 18 and 75 years. Most of the studies were performed in the combination of both genders (47–51), except two studies that performed in women and men separately (52, 53). Four studies were performed in the United States (47–49, 51), one in Germany (50), one in China (52), and one in Finland (53). The results of each of the studies by Batsis et al. (2018) (47), Zhao et al. (2017) (48), Min et al. (2017) (49), and Müezzinlera (2016) (50) were included as two separate studies as overweight and obese individuals; in addition, the study by Strandberg et al. (2011) (53) was included as two independent studies of those in the age range of 30–45 years and those in the age range of 75–85 years. In three studies (47, 49, 52), LTL in overweight or obese individuals was significantly lower than non-obese or non-overweight individuals. In addition, in two studies, (50, 53), LTL in obese/overweight was non-significantly lower than non-obese/non-overweight individuals. In two studies (48, 51), LTL was either significantly or non-significantly higher than the lowest category. The included studies’ characteristics are shown in Tables 1, 2. The OR of the association between shorter telomere length and obesity was only reported in two studies (54, 55); similarly, the comparison of body fat in different telomere length categories was only reposted in three studies (38, 40, 42); thus, because of the limited number of studies, no analysis was performed. Only one study provided the comparison of LTL among those with high body fat mass vs. those with low body fat mass (47); therefore, it was impossible to perform a meta-analysis.

**TABLE 1:** Characteristics of studies included in the systematic review owing to report the comparison of BMI between the lowest vs. the highest LTL categories.

First Author	Country	Journal	Study Population	Gender	Age	rTLT assay	Num.	Obesity/ overweight	Adjusted confounders	Main finding
Linghui (37)	China	Fron Aging Neurosci	Healthy	Both	65–80	qPCR	2,006	Obesity	Unadjusted	Non-significant lower BMI in the highest vs. the lowest rTLT categories (*P* = 0.585)
Zgheib (38)	Lebanon	Aging and Disease	Healthy	Both	> 18	qPCR	497	Central obesity	Unadjusted	BMI in the highest tertile of rLTL was significantly lower than the lowest (*P* = 0.045)
Milte (39)	Australia	Eur J Nutr	Healthy	Both	57–68	qPCR	679	Obesity	Unadjusted	Non-significant lower BMI in the highest vs. the lowest rTLT categories (*P* = 0.116)
Mazidi (40)	United States	Angiology	Healthy	Both	> 18	qPCR	8,892	Obesity	Age, race, sex	Non-significant lower BMI in the highest vs. the lowest rTLT categories (*P* = 0.312)
Mwasongwe (41)	United States	Atherosclerosis	Healthy	Both	> 21	qPCR	5,306	Obesity	Age, sex	Non-significant higher BMI in the highest vs. the lowest rTLT categories (*P* = 0.30)
Mazidi (42)	United States	Oncotarget	Healthy	Both	> 18	qPCR	5,020	Obesity	Unadjusted	BMI in the highest rLTL quartile (26.4 ± 0.21) was significantly lower than the lowest (28.5 ± 0.18) *P* < 0.001
Julin (43)	United States	Eur J Nutr	Healthy	Men	40–75	qPCR	2,483	Obesity	Age	BMI in the highest rLTL quartile (25.8 ± 3.2) was significantly lower than the lowest (26.2 ± 3.5) *P* = 0.05
Hardikar (44)	United States	BMC Obesity	Barrett’s esophagus	Both	50–70	qPCR	295	Obesity	Age, sex	BMI in the highest rLTL quartile (29.1 ± 4.3) was significantly higher than the lowest (28.1 ± 3.6) *P* = 0.05
Zalli (45)	United Kingdom	PNAS	Healthy	Both	54–76	qPCR	333	Obesity	Unadjusted	No significant difference between the lowest vs. the highest rTLT categories
Chen (5)	United States	Aging	Healthy	Both	30–50	qPCR	3,256	Obesity	Age	BMI in the highest rLTL quartile (30.1 ± 7.6) was significantly lower than the lowest (33 ± 7.6) *P* < 0.001
Liu (46)	United States	Am J Epidemilo	Healthy	Both	30–55	qPCR	4,604	Obesity	Age	BMI in the highest rLTL quartile (25.4.1 ± 4.5) was significantly lower than the lowest (25.8 ± 5) *P* = 0.03
Cassidy (4)	United States	Am J Clin Nutr	Healthy	Women	30–55	qPCR	2,284	Obesity	Age	BMI in the highest rLTL quartile (25.3.1 ± 4.3) was significantly lower than the lowest (26 ± 4.9) *P* = 0.005

**TABLE 2:** Characteristics of studies included in the systematic review owing to report the comparison of LTL between obese/overweight vs. non-obese/non-overweight individuals.

First author	Country	Journal	Study population	Gender	Age	rTLT assay	Num.	Obesity/overweight	Adjusted confounders	Main finding
Batsis (47)	United States	Int J Obes	Healthy	Both	> 18	qPCR	7,827	Obesity + overweight	Stratification by age	rTLT in overweight and obese individuals was significantly lower than those with normal weight (*P* < 0.001)
Zhao (48)	United States	Oncotarget	Healthy	Both	20–85	qPCR	12,792	Obesity + overweight	Age, gender	rTLT in obese was higher than overweight and normal weight individuals (*P* < 0.001)
Min (49)	United States	Eur J Nutr	Healthy	Both	> 20	qPCR	3,660	Obesity + overweight	Age, gender, ethnicity, income, smoking, alcohol, BMI, history of diabetes	rTLT in obese and overweight individuals was significantly lower than normal weight individuals (*P* < 0.001)
Müezzinlera (50)	Germany	Exp Gerontol	Healthy	Both	50–75	qPCR	3,600	Obesity + overweight	Age	rTLT in obese and overweight individuals was non-significantly lower than normal weight individuals (*P* = 0.074)
Cui (52)	China	obesity	Healthy	Women	40–70	qPCR	2,912	Obesity	Age	Those with the highest BMI had significantly lower rTLT compared with others (*P* = 0.005)
Strandberg (53)	Finland	J Gerontol	Healthy	Men	30–45	qPCR	480	Obesity	Age	rTLT in obese and overweight individuals was non-significantly lower than normal weight individuals (*P* = 0.06 and 0.07 respectively)
Fitzpatrick (51)	United States	Med Sci	Healthy	Both	> 65	qPCR	1,136	Obesity	Age	Non-significantly higher LTL in obese vs. non-obese individuals (*P* = 0.32)

*The results of each of the studies by Batsis JA et al. (47), Zhao H et al. (48), Min YB et al. (49), and Müezzinlera A (50) were included as two separate studies as overweight and obese individuals.*

*In addition, the study by Strandberg TE (54) was included as two independent studies of those in the age ranges of 30–45 years and those in the age range of 75–85 years. All of the included studies had cross-sectional designs.*

### Results of Meta-Analysis

The results of a two-class meta-analysis for the association between overweight/obesity and LTL are presented in Figure 2. The results showed that being in the highest category of LTL was associated with an approximate reduction of 0.75 kg/m^2^ in BMI (WMD = −0.75 kg/m^2^; CI = −1.19, −0.31; *p* < 0.001; *I*^2^ = 99.4%). The two-class meta-analysis of the comparison of LTL between overweight/obese vs. non-overweight/obese is presented in Figure 3; as it is shown, being overweight/obese was associated with a 0.036 kbp reduction in relative telomere length (WMD = −0.036; CI = −0.05, −0.02; *p* = 0.030; *I*^2^ = 100%). For finding the source of heterogeneity, subgrouping was performed, and the results are available in Tables 3, 4. Subgroupings showed that continent, age, and sample size could be possible sources of heterogeneity because of the slight reduction in heterogeneity after subgrouping according to these variables. The results of the quality assessment according to the AHRQ checklist (Supplementary Table 3) revealed that all of the studies had a moderate or high-quality score, and there was no study with poor quality. Among them, seven studies had moderate and twelve had high-quality scores. Publication bias was assessed with the funnel plots (Supplementary Figure 1). Moreover, Begg’s and Egger’s regression tests were further used to better clarify the publication bias. Accordingly, no evidence of publication bias was achieved for study parameters (BMI in the highest vs. the lowest relative telomere length categories: *p*_Egger_ = 0.131; *p*_Begg_ = 0.131; relative telomere length in overweight/obese vs. non-overweight/non-obese: *p*_Egger_ = 0.44; *p*_Begg_ = 0.41).

**FIGURE 2:** Weighted mean difference (WMD) with 95% confidence interval (CI) of the comparison of BMI in the lowest vs. the highest leukocyte telomere length.

**FIGURE 3:** Weighted mean difference (WMD) with 95% confidence interval (CI) of the comparison of leukocyte telomere length in obese vs. non-obese.

**TABLE 3:** Results of subgroup analyses of the comparison of BMI in those with the highest vs. the lowest relative telomere length (rTLT) according to the study or participants “characteristics”.

Group	No. of studies	WMD (95% CI)	*P*	P_heterogeneity_	I^2^, %	P_between study heterogeneity_
Total*	12	−0.75 −1.19, −0.31	0.001	< 0.001	99.4	
**Health status**						< 0.001
Apparently healthy	11	1.00 −0.11, 2.11	<0.001	< 0.001	99.5	
Patients with CVD risk factors, Barrett’s Esophagus	1	−0.87 −1.32, −0.42	0.077	−	−	
**Continent**						< 0.001
United States	8	−0.83 −1.33, −0.32	0.001	< 0.001	99.6	
Europe	1	−0.90 −1.92, 0.19	0.083	−	−	
Asia/Australia	3	−0.46 −1.75, 0.82	0.478	0.018	75.1	
**Sample size**						< 0.001
≤ 1,000	4	−0.49 −1.57, 0.58	0.364	0.016	71.1	
1,000–5,000	5	−0.74 −1.50, 0.02	0.056	< 0.001	89.8	
> 5,000	3	−1.009 −1.77, −0.24	0.010	< 0.001	99.9	
**Gender**						< 0.001
Both	10	−0.80 −1.28, −0.32	0.001	< 0.001	99.5	
Men or women	2	−0.48 −0.8, −0.17	0.003	0.403	0	
**Quality score**						< 0.001
5 ≥	3	−1.047 −2.853, 0.760	0.256	< 0.001	94.9	
5–9	7	−0.478 −1.177, 0.22	0.703	< 0.001	100	
≥ 9	3	−0.348 −2.138, 1.44	0.179	< 0.001	88.1	
**Age range**						< 0.001
> 18–20	4	−1.09 −1.80, −0.39	0.002	< 0.001	99.8	
30–75	6	−0.73 −1.49, −0.03	0.041	< 0.001	87.6	
> 65	2	0.081 −1.04, 1.20	0.888	0.135	55.3	

*Note that because all of included studies had cross-sectional designs, and the relative telomere length measurement method was quantitative polymerase chain reaction (qPCR); therefore, subgrouping according to these parameters was not performed.

**TABLE 4:** Results of subgroup analyses of the comparison of relative telomere length (rTLT) in obese vs. non-obese individuals according to the study or participants “characteristics”.

Group	No. of studies	WMD (95% CI)	*P*	P_heterogeneity_	I^2^, %	P_between study heterogeneity_
Total*	12	−0.036 −0.05, −0.02	<0.001	< 0.001	100	
**Weight status**						< 0.001
Obese	8	−0.042 −0.07, −0.014	0.003	< 0.001	99	
Overweight	4	−0.025 −0.058, 0.008	0.145	< 0.001	100	
**Continent**						< 0.001
United States	7	−0.019 −0.044, 0.005	0.127	< 0.001	100	
Europe	4	−0.076 −0.144, −0.007	0.03	< 0.001	94.5	
Asia/Australia	1	−0.013 −0.016, −0.010	< 0.001	−	−	
**Sample size**						< 0.001
≤ 1,000	2	−0.115 −0.223 −0.007	0.037	< 0.001	96.9	
1,000–5,000	6	−0.025 −0.031 −0.019	<0.001	< 0.001	96.8	
> 5,000	4	−0.020 −0.057 0.017	0.293	< 0.001	100	
**Gender**						< 0.001
Both	9	−0.022 −0.044 0.000	0.052	< 0.001	100	
Men or women	3	−0.080 −0.173 0.013	0.090	< 0.001	98.6	
**Quality score**						< 0.001
6 ≥	3	−0.041 −0.060 −0.022	<0.001	< 0.001	99.8	
8	2	−0.030 −0.031 −0.029	< 0.001	1	0	
9	7	−0.017 −0.027 −0.007	0.001	< 0.001	98.9	
**Age range**						< 0.001
> 18–20	6	−0.023 −0.049 0.002	0.071	< 0.001	100	
40–75	4	−0.063 −0.143 0.016	0.118	< 0.001	97.7	
> 75	2	−0.008 −0.125 0.108	0.889	0.014	83.5	

*Note that because all of included studies had cross-sectional designs, they were performed in healthy individuals, and the relative telomere length measurement method was quantitative polymerase chain reaction (qPCR); therefore, subgrouping according to these parameters was not performed.

## Discussion

The results of the current meta-analysis showed that those in the highest category of LTL had 0.75 kg/m^2^ lower BMI compared with those in the lowest category. Moreover, obese individuals had 0.04 kbp lower telomere length compared with non-obese. This study involved more than 35,655 adults in the age range of 18–80 years from different regions. In all of the studies, LTL was assessed with amplifying telomere and single-copy gene separately, using quantitative real-time polymerase chain reaction (RTqPCR), thus the results could be comparable, and this would minimize the possibility of measurement bias. After stratification of results according to the several confounders, in younger ages (<18–20 years old), there was a more pronounced reduction in BMI in the higher category of LTL rather than the lowest category. In addition, in stratification according to being overweight or obese, obese individuals had significantly lower (−0.042 kbp) telomere length, whereas this comparison was non-significant for overweight individuals. In the current study, we performed a two-class meta-analysis of the direct comparison of variables (either telomere length or BMI) in our case and control groups (either obese vs. non-obese or those with the highest vs. the lowest telomere lengths). This is a direct, more accurate, and robust representation of the study’s parameters compared with the meta-analysis of standardized regression coefficients that were performed in the previous meta-analysis of the association between BMI and telomere length by Gielen et al. (2018) (56); meta-analysis of regression coefficient is a controversial issue in the field of meta-analysis since it belongs to the regression models that include different sets of covariates and thus cannot be an accurate representation of the same parameter, and thus their direct combination is meaningless (57).

The association between LTL and obesity can be explained by several mechanistic pathways; first, obesity is a potent inducer of oxidative stress and inflammation, which increase the telomere shortening (58); obesity is associated with increased markers of oxidative stress including *malondialdehyde* (MDA), hydrogen peroxide, and reactive oxygen species (ROS), which can contribute to telomere shortening (56, 59–61). Numerous experimental and human studies revealed the role of oxidative stress in telomere shortening, telomere damage, and accelerating telomere attrition in a tissue-specific state (62, 63). It is established that chronic oxidative stress compromises telomere integrity (64, 65), and even telomere length shortening could be assumed as a biomarker of oxidative stress (66, 67). In addition, increased leptin concentrations in obesity, as an important pro-inflammatory adipokine, are associated with reduced LTL as revealed by Broer et al. (2014) in seven independent cohort studies of more than 11,448 participants (68). Moreover, the fat mass- and obesity-associated (*FTO*) gene is also another regulator of telomere length in obese individuals; this is done by two direct pathways of Fe (II)—and 2OG-dependent dioxygenase family and indirect method *via* expression of upstream/downstream flanking genes (69, 70). A summary of these mechanistic pathways is illustrated in Figure 4.

**FIGURE 4:** Mechanistic pathways of the possible role of obesity and obesity-related risk factors on leukocyte telomere length shortening.

From our stratified analysis given in Tables 3, 4, several findings were interesting: first, the negative association between BMI and telomere length was only pronounced and significant in the studies that were performed in the United States. The western diet that is more common in the United States is high in saturated fats and low in fiber, and omega-3 fatty acids can trigger telomere shortening; in a study by García-Calzón et al. (2015) (71), the high inflammatory potential of the diet was associated with shorter LTL among subjects with increased cardiovascular risk factors. In another study by Cassidy et al. (2010) (4), higher dietary fat and lower dietary fiber were associated with shorter telomere length. Moreover, the negative association between telomere length and BMI was more pronounced in younger ages; the possible explanation is that BMI is a more accurate measure of adiposity in younger ages compared with older adults because of loss of muscle mass in elderly (56). Since BMI is an indicator of general obesity and could not differentiate excess skeletal muscle from mass fat mass (72, 73), it is better to use other indicators of obesity (e.g., fat mass) with BMI. But as mentioned before, a very limited number of studies provided the results of fat mass (38, 42, 47); therefore, we could not provide the fat mass-related data here. It could be considered as one of the limitations of the current work.

## Conclusion

In conclusion, shorter telomere length was associated with higher BMI and obesity; this finding was different according to age and geographical distribution. Although the observational design of studies might limit the interpretation of causality, the stratification according to several confounders will increase the generalizability of the results. Given this, it is important to focus on the role of obesity in the aging process and further highlight the role of interventions to prevent against telomere shortening in obese individuals. Therefore, a meta-analysis of interventional studies regarding the prevention of telomere shortening in obesity is warranted.

## Data Availability Statement

The raw data supporting the conclusions of this article will be made available by the authors, without undue reservation.

## Author Contributions

SK and SH were involved in extraction of data, quality assessment, and writing the related parts in the manuscript. DB and TM were involved in manuscript English revision and data analysis and also wrote the related part of data analysis in the manuscript. SR was involved in manuscript revision, data analysis, and extraction and first articles’ screening. NN was also involved in first manuscript writing. MA-F supervised the project, generated the first idea, and hypothesis of work and was involved in manuscript revision. All authors read and agreed with final submission of manuscript.

## Conflict of Interest

The authors declare that the research was conducted in the absence of any commercial or financial relationships that could be construed as a potential conflict of interest.

## Publisher’s Note

All claims expressed in this article are solely those of the authors and do not necessarily represent those of their affiliated organizations, or those of the publisher, the editors and the reviewers. Any product that may be evaluated in this article, or claim that may be made by its manufacturer, is not guaranteed or endorsed by the publisher.
